# Effects of Puerarin Combined with PLGA/TCP/Puerarin on Osteocalcin and Sialoprotein of Mandibular Defects

**DOI:** 10.1155/2022/5177419

**Published:** 2022-09-06

**Authors:** Ying Guo, Qianqian Zhang, Nu Mi, Chunmei Li, Xuechao Lv, Hong Wang

**Affiliations:** ^1^Department of Stomatology, Shenzhen University General Hospital, Shenzhen 518055, China; ^2^Institute of Stomatological Research, Shenzhen University, Shenzhen 518055, China; ^3^Department of Stomatology, Shenzhen OCT Hospital, Shenzhen 518000, China; ^4^Department of Outpatient Stomatology, Heilongjiang Provincial Hospital, Harbin 150000, China; ^5^Department of Pediatric Dentistry, The First Affiliated Hospital of Harbin Medical University, Harbin 150000, China

## Abstract

In order to evaluate the effects of puerarin combined with poly lactic-co-glycolic acid (PLGA)/tricalcium phosphate (TCP)/puerarin on osteocalcin and sialoprotein of mandibular defects, the obtained rat jaw cells are analyzed. The surface morphology of osteoblast complex in the scaffold material group and puerarin combined scaffold material group is observed by a scanning electron microscope, and the growth and proliferation of osteoblasts are detected by the Cell Counting Kit-8 (CCK-8) method. Besides, the expression of type-I collagen (COL-I), osteocalcin (OC), and osteopontin (OPN) mRNA and related proteins in osteoblasts are detected by immunocytochemical staining. The results of immunocytochemical staining show that puerarin and PLGA/TCP/puerarin scaffold had significant effects on the expression of COL-I and OC mRNA and related proteins in osteoblasts. The experimental results indicate that puerarin and PLGA/TCP/puerarin can synergistically affect the mRNA and protein expressions of COL-I, OC, and OPN in osteoblasts and have a positive effect on promoting the proliferation activity of osteoblasts.

## 1. Introduction

Periodontitis is a chronic bacterial infectious disease that occurs in periodontal supporting tissue. Periodontitis causes tooth loosening and falling off, which seriously affects patients' oral health [1]. Periodontal pathogens not only cause direct damage to periodontal tissue through bacteria themselves and their toxic metabolites but also cause serious damage to the body through long-term persistent inflammation and immune response caused by bacteria [2]. As one of the common clinical problems in stomatology, periodontitis leads to alveolar bone absorption and jaw defects, which seriously affect the beauty, chewing, and pronunciation of patients [3]. The classic method of clinical treatment of alveolar bone and jaw defects is to use appropriate bone filling materials to fill the defect site, so as to enhance the ability of defect repair. At present, bone tissue engineering technology provides a good prospect for the reconstruction of personalized and functional bone defects in the repair of jaw defects. However, there are still many deficiencies in biomaterials [4]. The emergence of 3D printing technology provides a new solution [5]. It realizes the construction of bioactive scaffolds to promote the bone through the function-oriented design of bone repair material structure and the manufacture of fine bionic structures with appropriate mechanical strength [6, 7]. It is also a hot topic of joint exploration in clinical oral and maxillary and biomaterial fields in recent years. In this study, the periodontitis model is established in rat maxillary molars and the jaw defect model is established in the mandibular body. A low-temperature 3D printing technology is used to combine the clinical drug puerarin into degradable polymer and bioceramic materials, and degradable porous drug-containing scaffold materials can be obtained eventually. To realize the effective repair of the inflammatory alveolar bone defect, the precise control of the molding process, good biocompatibility, appropriate mechanical properties, controllable microporous structure, controllable degradation rate, and the growth rate of new bone roughly should be collaborated synchronously.

The rest of the study is organized as follows: Section 2 discusses related studies, and Section 3 introduces the experimental materials and proposed methods.  Section 4 describes the comparative results and analysis chiefly.  Section 5 provides the summary.

## 2. Related Works

Maxillofacial trauma, inflammation, tumors, and other diseases can cause jaw defects, which often lead to facial deformities and masticatory dysfunction [8]. However, the complex shape and function of the jaw is a major challenge for maxillofacial surgery [9]. With the continuous development of immunology, material science, cell biology, and tissue engineering, new materials, new technologies, and new methods emerge in endlessly. The rise of tissue engineering provides more theoretical guidance and technical support for the treatment of jaw defects. Osteoblasts and biological scaffold materials are important elements in bone tissue engineering [10, 11].

The participation of cells is very important in tissue engineering bone construction. In the case of a large bone tissue defect, if there are not enough osteoblasts around the bone repair material, the bone cannot be formed [12]. In cavity-type bone defects, the wound surface is lined with a large amount of blood and tissue fluid, containing a large number of undifferentiated mesenchymal cells. There are also a large number of osteoblast precursors on the wound surface of the bone, and these cells with osteogenic potential can enter the gap of the repair material and fill the whole bone repair area and then proliferate and differentiate into the new bone under the biological induction of the material [13, 14]. The PLGA/TCP/puerarin scaffolds can overcome not only the defects of biocompatibility, biodegradability, and bone tissue engineering orientation of previous materials but also have the characteristics of other materials that are difficult to solve the category of osteogenic activity with existing theories. To screen the gene spectrum and express the induction factor required for tissue creation, for instance, the ideal proportion combination of a variety of inorganic active components in the material can be used. [15]. The specific surface area is large, and there are numerous nanopores that are beneficial to cell proliferation and formation of new tissues. It has significant gene regulation effects on calcifying elements such as osteocalcin and alkaline phosphatase [16]. It has a compound three-dimensional structure with a specific proportion of inorganic active elements and a porosity of over 90%, which enables it to adhere to and accommodate osteoblasts and chondrocytes and microvascular and regulate osteoblasts, thereby releasing bone growth factors and inorganic elements in a specific proportion. At the same time, inorganic elements released during the degradation of scaffold materials can provide nutritional channels necessary for the survival of living cells by neutralizing the acid decomposition products of polylactic acid with its weak alkalinity. Large bone tissue defects can be repaired quickly and effectively by a biological combination of direct central mineralization and osteogenesis [17].

As an isoflavone compound, puerarin has the effects of slowing down heart rate, dilating blood vessels, and lowering blood pressure. It is mainly used in the treatment of hypertension, angina pectoris, cerebral insufficiency, and cerebral infarction [18, 19]. Due to the preventive effect on osteoporosis, extensive attention of researchers has been attracted recently. Some studies have found that puerarin can promote the proliferation and differentiation of osteoblasts, improve alkaline phosphatase activity, and have a good stimulating effect on alkaline phosphatase activity through in vitro culture of human osteoblasts, which may indicate that puerarin has the function of improving osteoblast bone formation [20, 21]. Scanning electron microscope observation showed that puerarin extended osteoblasts well on PLGA/TCP/puerarin repair scaffold, could be connected into sheets, cell matrix secretion is normal, cells and cell matrix could cover the surface of the material, and had good biological compatibility. PLGA/TCP/puerarin repaired scaffolds can also promote the rapid proliferation of osteoblasts.

Type-I collagen (COL-I), osteocalcin (OC), and osteopontin (OPN) are important osteogenic factors and markers of osteoblast differentiation. Col-I, specific collagen secreted by osteoblasts, is the main bone structural protein, providing a scaffold for calcium salt deposition and cell adhesion and can be used as an indicator to evaluate the functional status of osteoblasts [22]. OC is a kind of noncollagenous protein specifically secreted by osteoblasts, which is a marker of osteoblast mineralization to the matrix and can reflect osteoblast activity. OPN is also one of the markers of osteoblasts [23]. OPN promotes the absorption and mineralization of the bone matrix and plays an important role in the process of bone formation and remodeling. In this study, mRNA and protein expressions of osteogenic factors COL-I, OC, and OPN in osteoblasts are detected by RT-PCR and immunocytochemical staining. COL-I, OC, and OPN proteins are all expressed in the cytoplasm of osteoblasts, and the positive reaction is brownish yellow granules. Factorial variance analysis shows that puerarin and porous tantalum scaffolded can synergistically promote the expression of COL-I and OC in osteoblasts. However, it has no significant effect on the expression of OPN. Previous studies have found that puerarin and estradiol can increase the expression of BSP and OCmRNA. Puerarin and estradiol can reduce the expression of OPNmRNA, suggesting that puerarin can promote osteoblast differentiation by affecting the mRNA expression of characteristic proteins related to osteoblast differentiation [24]. Other studies found that puerarin significantly increased ALP activity and COL-I secretion within 0.01∼1 *μ*mol/L in a dose-dependent manner to promote differentiation and maturation of human osteoblasts [25].

## 3. Experimental Materials and Proposed Methods

### 3.1. Study Objects

3-4-week-old female SD rats, SPF grade, were supplied by Shanghai Slack Experimental Animal Center; the primers for OPG, RANKL, Runx2, OPN, OC, and GAPDH are synthesized by Shanghai Shenggong Bioengineering Co., Ltd. Gegensu is purchased from Shanghai Hengfei Biotechnology Co., Ltd. (Art. P9050); DMEM high sugar medium is purchased from Shanghai Microscience Biotechnology Co., Ltd. (Art. L0104-100). SDS-PAGE gel preparation kits (LPS, FBS, PBS buffer, Trypsin-EDTA digestive solution, 100 × penicstreptomycin mixture) are purchased from Solarbio, Inc. ((Art. L8880, 11011–8611, P1022, T1300, P1400, P1200-) 50 t); osteogenesis induction medium is purchased from Baizhi Biomedical Technology (Shanghai) Co., Ltd. (Biosmedi-DF-8001). RNAiso Plus, reverse transcription kit, and fluorescence quantitative PCR kit are purchased from Takara Company in Japan (article number: RR037Q/A/B, 639519). Alkaline phosphatase detection kit, RIPA lysate, and BCA kit are purchased from Shanghai Biyuntian Company (article number: P0321, P0013 K, P0011). 3900 high throughput DNA synthesizer is purchased from Applied Biological Systems, Inc. CFX96 Touch Deep Well Fluorescent quantitative PCR instrument is purchased from Bio-Rad Company, USA. Elx800 microplate meter, 1659001 protein electrophoresis meter, and Trans-Blot SD semidry membrane transfer instrument are purchased from Bio-Rad Company in the United States. The Ckx41-f32f optical microscope is purchased from Olympus Company, Japan. Centrifuge 5424R low-temperature high-speed centrifuge is purchased from Eppendorf GMBH in Germany.

### 3.2. Main Reagents and Instruments

#### 3.2.1. Isolation and Culture of Rat Jaw BMSCs

The female SD rats aged 3-4 weeks are sacrificed by neck dissection and immersed in 75% ethanol solution for 5 min. The mandible and bilateral iliac bones are removed, respectively, in a sterile environment, the attached soft tissues are removed, and sterile PBS is repeatedly rinsed. Next, the bone marrow puncture needle 21# is used to pierce 4-5 holes in the bone cortex, and the cells are repeatedly rinsed with *α*-DMEM. The collected cell suspensions are placed in Petri dishes and cultured at 5% CO_2_ and 37°C. After 48 h of culture, BMSCs are first half-changed and then the fresh medium is replaced every 3 days. The proliferation number and growth status of stem cells are observed by an inverted phase contrast microscope. The third-generation BMSCs can be used for the experiment.

#### 3.2.2. Preparation of Complete Medium

Add 10% fetal bovine serum and 100 U/mL penicstreptomycin into DMEM high-glucose medium and mix them upside down. The purchased frozen cell lines are thawed in a waterbath at 39°C for 1000 r/min, centrifuged at room temperature for 5 min, suspended in a complete medium, mixed, and cultured in a cell incubator with 5% carbon dioxide at 37°C. When the cells grew to about 85%, the cells are digested with trypsin and subcultured in a 96-well plate at a ratio of 1:3. Mc3t3-e1 cells are divided into the control group, model group, and puerarin group by the random number table method. Mc3t3-e1 cells are treated with 1 µg/mL LPS for 24 h. The puerarin group cells are treated with 10 nmol/L puerarin (dissolved in DMEM high sugar medium) and cultured for 24 h. Cells of each group are collected on three plates for reserve, and the cell culture medium of each group is collected on the other plate. After being rinsed by PBS, cells are fixed with 4% paraformaldehyde solution for reserve.

#### 3.2.3. Cells Are Cocultured with Puerarin Combined with PLGA/TCP/Puerarin Scaffold Material

PLGA/TCP/puerarin scaffold material is cleaned with ultrasonic cleaner for 15 min and autoclaved for 30 min. It is then kept into a sterile 6-well plate, *α*-MEM medium prewet, and 24 h later, the excess liquid is discarded andset aside. 300 *μ*L 1 *μ*mol/L drug-treated cell suspension with a density of 2 × 10^4^ cells/mL is inoculated on the surface of scaffold material and incubated at 37°C for 2 h in an incubator with 5% CO_2_. The scaffold material is turned upside down and the other side of the material is added according to the above inoculation method and incubated at 37°C for 2 h in an incubator with 5% CO_2_. 2 mL *α*-MEM medium is added into each well, and the culture is continued.

#### 3.2.4. Experimental Grouping

The scaffold material group is defined as PLGA/TCP/puerarin scaffolds that are cocultured with osteoblasts. Puerarin combined with the scaffold material group is defined as puerarin, PLGA/TCP/puerarin scaffold materials that are cocultured with osteoblasts. Besides, the blank group is defined as osteoblast culture.

### 3.3. Detection of Osteogenic Differentiation

#### 3.3.1. CCK-8 Method

A 50 *μ*L CCK-8 solution is added, and the 24-well plates are placed in an incubator with 5% CO_2_ at 37°C for 2 h. Absorb 100 *μ*L supernatant from each well of the 24-well plate and add it successively to each well of the 96-well plate. The absorbance (OD) of each well in the 96-well plate is measured by a microplate reader at 490 nm.

#### 3.3.2. Expression Levels of COL-I, OC, and OPNmRNA Are Detected by RT-PCR

Trizol's one-step method is used to extract the total RNA from each group of osteoblasts cultured for 5 days. The total RNA concentration and purity are calculated according to the formula, and the RNA concentration is adjusted to 500 ng/*μ*L. CDNA is synthesized using M-MuLV reverse transcriptase, Primer5.0 software is used to design primers, and PCR primer sequences of each gene are synthesized, as shown in Table 1. SYBRqPCRMix is used for PCR amplification system reaction. The PCR amplification system is set to reverse for 5 s, annealing at 56°C for 25 s, extension at 72°C for 20 s, a total of 40 cycles, and extension at 72°C for 5 min. PCR results are analyzed using Comparative delta-delta Ct.

#### 3.3.3. Expression of COL-I, OC, and OPN Proteins by Immunocytochemical Staining

Each group is prepared into single-cell suspension and inoculated into a 6-well plate with sterile cover glass at a density of 1 × 10^6^ cells/mL. After the cells grew to semiconglutination, the sterile cover glass is taken out, ished with PBS 3 times, fixed with 4% paraformaldehyde for 30 min, discarded paraformaldehyde solution, and ished with PBS 3 times; an appropriate amount of 0.5% Triton-100 is dropped onto the cover glass, which is lysed at room temperature for 20 min, and ished with PBS 3 times, 2 min per time. An appropriate amount of 3% of H_2_O_2_ is dropped onto the cover glass and incubated at room temperature for 15 min to achieve the effect of blocking endogenous peroxidase, and ished with PBS 3 times and added a proper amount of primary antibody (1:150)overnight at 4°C, ished with PBS 3 times, 2 min/time; an appropriate amount of secondary antibody is dropped and incubated at 37 °C for 30 min and then ished 3 times with PBS, 2 min each. DAB is used for color rendering, and the cover glass is immersed in gradient alcohol for step-by-step dehydration. Xylene is transparent, and neutral gum is used for routine sealing. Image-Pro Plus Image analysis software is used for semiquantitative analysis of dyeing index results.

### 3.4. Observation Indicators

The observation indicators include the following: (1) PLGA/TCP/puerarin scaffold materials and composites are observed under scanning electron microscopy; (2) observe the proliferation of osteoblasts; (3) the mRNA expression levels of COL-I, OC, and OPN in osteoblasts are observed; (4) the expressions of COL-I, OC and OPN proteins in osteoblasts are compared.

### 3.5. Statistical Treatment

SPSS 26.0 software is used for statistical analysis of the data, and the count data are expressed as rate (%). The mean ± standard deviation of measurement data indicated that one-way ANOVA is performed for comparison between groups, and the LSD *t*-test is used for further pairwise comparison. *P* < 0.05 is considered statistically significant.

## 4. Comparative Results and Analysis

### 4.1. Scaffold Materials and Composites under Scanning Electron Microscopy

The PLGA/TCP/puerarin scaffold material under scanning electron microscopy has a large number of uniformly dispersed microporous structures with diameters of about 400∼600 *μ*m. The internal pores are interconnected, and the interpore trabecular pillars are microporous. Under scanning electron microscopy, osteoblasts are observed on the surface of the scaffold material and in the micropores to form layers of adhesion and growth, extending out cell pseudopodia, connecting with each other, and fusing into sheets, and secreted matrix covered the surface of the scaffold and in the micropores. The results showed that osteoblasts had good extensibility on the scaffold and could be connected into sheets. The secretion of the cell-matrix is normal, and cells and cell matrix could cover the surface of the scaffold material, as shown in Figure 1.

### 4.2. Observation of the Proliferation of Osteoblasts

OD values of each group are measured at 1 d, 3 d, 5 d, and 7 d by ELISA. The results indicate that the proliferation activity of puerarin combined with the scaffold material group increased significantly than that of the blank group with the time extension, with a statistical significance (*P* < 0.05). The proliferation activity of the scaffold material group increases significantly than that of the blank group (*P* < 0.05), as shown in Table 2. The symbol “*∗*” represents *P* < 0.05 compared with the blank group.

### 4.3. Comparison of the mRNA Expression Levels of COL-I, OC, and OPN in Osteoblasts

In this experiment, the CT method is used to analyze and process the data, and it is shown that the mRNA expression levels of COL-I and OC in puerarin combined with the scaffold material group and scaffold material group increased significantly than those in the blank group (*P* < 0.05), and the mRNA expression levels of COL-I and OC in puerarin combined with the scaffold material group increased significantly than those in other groups. There is no significant difference in the expression of OPN mRNA among all groups (*P* > 0.05). After one-factor analysis of variance, puerarin and PLGA/TCP/puerarin scaffold materials can promote the high expression trend of COL-I and OC mRNA in osteocytes. The expression of COL-I and OC mRNA is synergistically promoted, but OPN mRNA is not significantly affected, as shown in Table 3. The symbol “#” represents *P* < 0.05 compared with the stent material group.

### 4.4. Expressions of COL-I, OC, and OPN Proteins in Osteoblasts

Analysis of osteoblasts in each group by immunocytochemical staining showed that COL-I, OC, and OPN proteins are all expressed in the cytoplasm of osteoblasts, and the positive reaction is brownish yellow granules, indicating that COL-I, OC, and OPN are expressed in different degrees in each group. The expression levels of COL-I and OC in the scaffold group are significantly higher than those in the blank group (*P* < 0.05), and the expressions of COL-I and OC in the puerarin combined with the scaffold group are significantly higher than those in the other groups (*P* < 0.05), but the comparison of OPN protein expression among all groups is *P* > 0.05. The results of one-way variance analysis show that puerarin and PLGA/TCP/puerarin scaffold materials can promote the expression of COL-I and OC proteins. They have a synergistic effect on the expression of COL-I and OC proteins but cause no significant effect on the expression of OPN protein, as shown in Table 4.

## 5. Conclusions

In this study, the effects of puerarin PLGA/TCP/puerarin repair scaffold on the expression and cell proliferation of osteoblast osteogenic factors COL-I, OC, and OPN are investigated. The experimental result can provide a scientific theoretical basis for puerarin and PLGA/TCP/puerarin repair scaffold materials for the treatment of bone defects and fracture healing. In addition, the medicinal value and clinical trial range of puerarin will be expanded based on the inherent clinical treatment of osteoporosis. The findings can improve the application scope of *Pueraria lobata* and play an important role in mining the medicinal value and economic value of *Pueraria lobata*. Isomorphism is an active attempt and exploration of the molecular biology experiment of traditional Chinese medicine. It can also bring positive exploration and attempt to the treatment of bone repair with integrated traditional Chinese and Western medicine. In future work, we will further explore the clinical effect of puerarin as an auxiliary drug for bone graft scaffold material to repair bone defects in promoting bone growth, so as to provide a theoretical and practical basis for further clinical application.

## Figures and Tables

**Figure 1:** Surface morphology of scaffold material and osteoblast complex is observed under the scanning electron microscope: (a) microporous structures; (b) S-4800 5.0 kV 15.5 mm × 1.00 (k) SE (M); (c) S-4800 5.0 kV 16.6 mm × 200 SE (M); (d) S-4800 5.0 kV 16.9 mm × 100 SE (M).

**Table 1:** Primers of target gene and reference gene.

Name of the primer	Primer	The sequence (5′-3′)
OC	Primer *F*	CCTTCATGTCCAAGCAGGA
	Primer *R*	GGCGGTCTTCAAGCCATAC

OPN	Primer *F*	GCTTGGCTTATGGACTGAGG
	Primer *R*	GGCTTTGGAACTTGCTTGAC

COL-1	Primer *F*	AGTGGTTTGGATGGTGCCAA
	Primer *R*	GCACCATCATTTCCACGAGC

GAPDH	Primer *F*	AGTCAGGTATCCCACAGGAAACAG
	Primer *R*	TGTGTCCGTCGTGGATCTGA

**Table 2:** Comparison of osteoblast proliferation (OD).

Group	1 d	3 d	5 d	7 d
The blank group	0.163 ± 0.035	0.425 ± 0.038	1.133 ± 0.047	1.351 ± 0.073
Bracket material group	0.177 ± 0.028^*∗*^	0.647 ± 0.031^*∗*^	1.161 ± 0.036^*∗*^	1.552 ± 0.051^*∗*^
Puerarin combined with the scaffold material group	0.179 ± 0.016^*∗*^	0.752 ± 0.046^*∗*^	1.184 ± 0.041^*∗*^	1.771 ± 0.046^*∗*^
F	1.134	4.276	4.023	5.117
*P*	0.112	<0.001	<0.001	<0.001

**Table 3:** Comparison of mRNA expression of COL-I, OC, and OPN in osteoblasts.

Group	COL-I	OC	OPN
The blank group (*n* = 3)	1.00	1.00	1.00
Bracket material group (*n* = 3)	1.45 ± 0.55	1.55 ± 0.25	1.08 ± 0.31
Puerarin combined with the scaffold material group (*n* = 3)	1.96 ± 0.27^*∗*^^#^	1.84 ± 0.59	1.14 ± 0.53
*F*	8.227	8.695	2.034
*P*	<0.001	<0.001	0.116

**Table 4:** Comparison of COL-I, OC, and OPN protein expression detected by immunocytochemical staining.

Group	COL-I	OC	OPN
The blank group (*n* = 9)	14.167 ± 0.525	16.215 ± 1.037	15.887 ± 0.664
Bracket material group (*n* = 9)	16.785 ± 0.872	17.526 ± 1.121	16.262 ± 1.427
Puerarin combined with the scaffold material group (*n* = 9)	18.221 ± 0.514	19.117 ± 1.134	16.354 ± 0.421
F	7.546	8.014	1.817
*P*	<0.001	<0.001	0.235

## Data Availability

The data used to support the findings of this study are available from the corresponding author upon request.
